The article "Urban Air Pollution and Greenness in Relation to Public Health" was published in 2023. Journal: J Environ Public Health.

# Urban Air Pollution and Greenness in Relation to Public Health

**DOI:** 10.1155/2023/8516622

**Published:** 2023-01-30

**Authors:** Addis Bikis

**Affiliations:** Mizan-Tepi University, Tepi, Ethiopia

## Abstract

**Background:**

Air pollution is the result of economic growth and urbanization. Air pollution has been progressively recognized as a serious problem for cities, through widespread effects on health and well-being. There is less concern from stakeholders about greenness and air pollution mitigating factors in an urban area. This research targeted to indicate the spatial dissemination of greenery, air quality levels (PM_2.5_, PM_10_, CO_2_, and AQI), and exposure to air quality-related health risks for the people in the urban area.

**Method:**

The data were collected by measuring air quality at transportation stations and manufacturing industries with Air visual pro, then observing and mapping greenness in the city within the administrative boundary by GIS (street greenery, forest, availability of greenness in the manufacturing industry), and lastly questionnaire and interview were employed for air quality-related health issues. Then, the air quality data were analyzed by using USAQI standards and health messages. Both quantitative and qualitative research approach had employed to explore air pollution levels, availability of greenness, and air quality-related health issues. Moreover, Health questionnaires and greenness were correlated with air quality levels by a simple linear regression model.

**Result:**

The result indicated that there was unhealthy air quality in the transportation and manufacturing industries. The measured air quality showed in a range of 50.13–96.84 *μ*g/m^3^ of PM_2.5_, 645–1764 ppm of CO_2,_ and 137–179 Air quality index (AQI). The highest mean of PM_2.5_ and air quality concentrations at Addis Ababa transportation stations and manufacturing sites ranged between 63.46 and 104.45 *μ*g/m^3^ and 179–326, respectively. It was observed with less street greenery and greenness available in residential, commercial areas, and manufacturing industries. The pollution level was beyond the limit of WHO standards. The result has shown a health risk to the public in the city, particularly for drivers, street vendors, and manufacturing industry employees. Among 480 respondents, 57.92% experienced health risks due to air pollution by medical evidence.

**Conclusion:**

High health risks due to industries and old motor vehicles in the city need to be reduced by introducing policies and strategies for low-carbon, minimizing traveling distance, encouraging high occupancy vehicles, and promoting a green legacy in the street network and green building.

The article "Urban Air Pollution and Greenness in Relation to Public Health" was published in 2023. Journal: J Environ Public Health.

## 1. Introduction

Globally, urban air pollution is a major concern. Air pollution is growing and has a negative impact on human health. Respiratory health diseases and social inequality have increased due to air pollution and the COVID-19 pandemic [1, 2]. In connection with this, greenness has been affirmed to decrease air pollution and improve quality of life [3, 4]. It has believed that reducing exposure to air pollution through greenness could improve the health of urban residents (Li et al., 2016; [5]. However, the available evidence on the effect of greenness on urban air pollution and the protection against COVID-19 has been inadequate and flexible. Air pollution is increasing due to rapid urbanization, the manufacturing industry, and carbon emission. This has caused for depleting green natural environment and underestimated the impact of the COVID-19 pandemic in undeveloped nations [6, 7]. Urban air pollution causes health problems especially, respiratory and cardiovascular diseases. According to research studied by Bikis and Pandey [8] in Addis Ababa, 40% of urban residents have been affecting health risks by transport-related air pollution. Moreover, there are many causes of urban air pollution, i.e., manufacturing, combustion engines, motor cars, cooking firewood, the construction industry, and dust. These sources emit poisonous gases into the atmosphere such as particulate matter (PM_2.5_), CO_2_, CO, SO_2_, NO_X_, and PM_10_.

Lockdown brought on by COVID-19 decreased economic and transportation activity, lowering energy use, and oil demand. The environmental quality is significantly impacted by these changes [9, 10]. Industries, transportation networks, and all other businesses have closed, and air pollution levels in New York, China, and India have all dropped by 50%, 25%, and 30%, respectively [11]. Carbon emissions have suddenly decreased as a result of this.

Overwhelming influences of urban air pollution on human health stays to rise. Reducing urban air pollution has become one of the key challenges faced by policymakers internationally [12, 13]. For this, the promotion of green infrastructure (GI) is considered a win-win solution to air pollution. It diminishes surface concentrations without imposing restrictions on traffic and other polluting sources [14–16].

Air pollution has become the main threat to human health. The United Nations Environmental Program has projected that 1.1 billion people breathe in unhealthy air globally [17]. Epidemiological studies have shown that the concentrations of airborne particles in the surrounding are associated with several human health effects, especially on the cardiovascular and respiratory systems [18]. The World Health Organization [19] has estimated that urban air pollution kills about 800,000 people, and 4.6 million people lost their survival worldwide every year. Therefore, the correlation between air pollution and exposure risk has been affecting the population's economy and health during the COVID-19 pandemic through increased treatment costs and access to quality healthcare [5, 20].

The article "Urban Air Pollution and Greenness in Relation to Public Health" was published in 2023. Journal: J Environ Public Health.

Ethiopian ministry of health reported that greater than 800,000 people have been affected by the respiratory disease in Addis Ababa four years ago due to air pollution. Agreeing with the air quality survey studied two years ago in 2019, ensuring that the air pollution level in Addis Ababa has become over the restriction ratified by the world health organization of 25 *μ*g/m^3^ of PM_2.5_ (WHO, 2011). Among 819,900 all patients who visited health institutions, 27.2% of them had been patients exposed to respiratory illness. According to WHO air quality rules and regulations, fine particulate matter pollution must not be greater than 20 *μ*g/m^3^. However, the number exceeded 300 *μ*g/m^3^ in some parts of Addis Ababa (Ministry of Health, 2018). Twenty leading respiratory and cardiovascular patients have visited health institutions in Addis Ababa [21]. These incidences of respiratory infection were the primary concern. This liked with the poisonous emissions of the transportation cars and manufacturing industry. Accordingly, in a study depicted by Tiwari [21] and Bikis and Pandey [8], acute respiratory infections were about 148,000 in 2007 and reached 207,000 in 2008 and 856,000 in 2019.

Middle-aged, children, and older people are also exposed to air pollution caused by CO_2_ and PM_2.5_ [22], which causes premature death [23] and raise the threat to health due to long-term respiratory illness [24]. The reported associations among increased respiratory, cardiovascular mortality, and chronic exposures to particulate matter were the highest [25, 26].

Many structures and development plans have been prepared at different times including implementation strategies for urban greenery and street trees to reduce urban air pollution and urban heat island. The city government and influential stakeholders have not given critical attention to greenery and street trees rather than consume infill development for the construction of buildings and roads. Because of this, air pollution has been rapidly increasing and affecting human health and the atmosphere in the city [13].

The industries are unregulated since the lack of proper social and environmental quality protection. Priority has only been given to economic development, but air quality concerns have been given less attention [12]. The emissions of industries have still currently not been controlled in Ethiopia. So, manufacturing industries remain to emit pollutants into the urban environment without any management, which has serious health and social consequences for people exposed to asthma and related diseases [27]. Moreover, air pollution has continued with less concern [4]. This is a common assumption by stakeholders that air pollution levels are below the risk zone and is not supported with practical evidence. Unavailable devices for measuring air quality inside the home and outside the urban environment in Ethiopia cities have increased exposure to health problems without management. Besides, the Environmental Protection Authority (EPA) and the Environmental Protection Bureau of the Addis Ababa City Government have not had sufficient documentation on the scope of the issue. In general, the existing land use of Addis Ababa city, especially the manufacturing industry, educational institution, and transportation terminals/stations, does not have sufficient greeneries and street trees. Therefore, this study investigated air pollution levels by air visual pro and green cover in relation to public health in Addis Ababa, Ethiopia.

The article "Urban Air Pollution and Greenness in Relation to Public Health" was published in 2023. Journal: J Environ Public Health.

## 2. Literature Reviews

### 2.1. Air Pollution and Sources

Pollution is defined as the release of substances dangerous to people and other living organisms into the environment [28]. Contaminants are hazardous solids or gases that are created in greater than normal concentrations and affected the quality of the environment [26]. Rapid urbanization and increasing transport consumption are inspired by population growth and increased economic activities in the city center [29]. Emission from various sources such as industry, old vehicles, dust, and cooking firewood deteriorate air quality and causes health problem for individuals (MohdShafie et al., 2022). Air pollution in Ethiopia is mainly produced by vehicles, followed by industries and domestic emissions. Monitoring air pollution has permanently been a challenge in low- and middle-income countries [30]. The growing number of cars led to more use of hydrocarbons such as petrol and emitting CO_2_ and PM_2.5_ into the atmosphere [31]. This contributes to the increase in emissions, which is the main source of the deterioration of air quality [32].

The implementation of green infrastructure by administrations and concerned bodies mainly reduces air pollution problems, specifically in the urban region. Urban greenery is important for many health benefits and ecosystem services. The leaves act as a -biofilter for particulate matter and pollutant gases and reduce air pollution in urban areas [33, 34].

The article "Urban Air Pollution and Greenness in Relation to Public Health" was published in 2023. Journal: J Environ Public Health.

An increasingly promoted way to mitigate air pollution is the use of green infrastructure, street greenery, green walls, green building [35], and familiarizing plantations into the urban landscape [36].

Having reviewed several studies conducted on urban air pollution, it was found that the concentration stages of the fine particulate matter (PM_2.5_) were 280 *μ*g/m^3^ in Addis Ababa [8]. Carbon monoxide (CO) levels were too greater than the recommended limit for public safety. Urban residents are using biomass fires in their favor that increases the air pollution level [37]. It is believed that more than 95% of most urban residents still want the traditional stove for cooking. This is a significantly increasing number of carbon dioxide (CO_2_). This was also documented in some random samples in the household home [38]. The majority of the samples collected were particulate matter levels above WHO guidelines. Randomly measured carbon monoxide (CO) levels alongside the city's roads were also higher than expected, despite an average yearly growth in car ownership growing by 9% [39].

Air pollution is a difficult issue in low- and high-income nations with considerable differences between the two in terms of causes and sizes [40]. In high-income countries, air pollution comes mostly from manufacturing and automotive sources since homes use clean fuel sources for cooking often electricity [17]. In low-income nations, air pollution is compounded due to the traditional use of solid biomass and mixed liquid fuels [4]. These toxic fuels are used in homes where females spend more time than males [41].

Indoor air pollution was studied much further in Addis Ababa city than that outdoor air pollution. Many studies show results based on the type of fuel used for cooking, rather than the actual number obtained by measurement. Researchers searched for PM_2.5_, nitrogen dioxide (NO_2_), polycyclic aromatic hydrocarbon (PAH), carbon monoxide (CO), and sulfur dioxide (SO_2_).

In 2012, measurement was taken over a 24-hour period at 59 homes in slum neighborhoods [41], the average value of PM_2.5_ was 1,134 *μ*g/m^3^. This is mainly used from solid biomass. The research conducted in the Oromia region found that household suspended particulate matter was 130 times more than that of the recommended air quality standards [42, 43]. This shows a serious health risk to the general public. Moreover, additional research was conducted in 10 Addis Ababa households that focused on the inhaling smoke produced from heated coffee beans and charcoal during a cultural ceremony. This study showed high PM exposure, with a mean of 1000 *μ*g/m^3^ PM concentration. This traditional coffee ceremony, which contains inhaling the smoke of burning coffee beans, is a small but frequent home activity that takes place 2–3 times per day [44].

The article "Urban Air Pollution and Greenness in Relation to Public Health" was published in 2023. Journal: J Environ Public Health.

### 2.2. Traffic and Road Conditions

According to the ministry of health [45], 60% of urban air pollution is caused by vehicle emissions. Many inhabitants of Addis Ababa city are living in the region where urban smoke, particle matter, CO, and CO_2_ from transport and road dust are causing severe health problems. Research conducted by Bikis and Pandey [8] has shown that recent plans for spatial location and design of transport stations do not consider the exposure of air pollution for waiting passengers. Due to this, the air quality has become a problem in the city. According to Gebre et al. [46]; the mass concentrations of total suspended particulate matter (PM_10_) in the city were found beyond the level of 150 *μ*g/m^3^.

The rate of vehicular increase in the city exceeds the volume of the road network that is being built. About 62% of the country's vehicles are found in the city of Addis Ababa [47]. The number of vehicles is growing by 9.88% each year, while the road networks are growing at a yearly growth rate of 8.22% [48]. Addis Ababa exposes a rise in air pollution due to the increasing number of automobiles which do not follow emission standards set by various environmental authorities. Subsequently, a study has shown that 53.5% of vehicles were above 20 years old, while 29.3% were above 30 years old [21]. This figure shows tailpipe emissions from the exhaust system. The main pollutants include carbon dioxide (CO_2_), particulate matter (PM), and sulfur dioxide (SO_2_) [39, 49]. There was no tangible information available to evaluate the particulate matter emissions for fuels with the different extents of biofuels.

### 2.3. Urbanization, Manufacturing, and Construction Industry

Rapid urbanization is a universal trend that impacts society and the environment. It is widely recognized that the majority of the global population lives in the urban region [50]. In 2014, a projected 54% (about 3.8 billion population) is living in the urban area [51]. 66% of the population is expected to live in cities by 2050, with the highest urban growth rates in low-income countries [52]. Rapid growth has caused suburban sprawl i.e., the unlimited growth of high-rise buildings, industries, services, and roads [4]. Urban sprawl is usually related to longer commutes and adds to traffic congestion and increased air pollution [53].

World Health Organization [16] report has shown that Ethiopia has the top road mortality rate per vehicle in the world. Roads in Ethiopia are poorly maintained, with poor signs and lighting [54]. In addition, the industry is contributing to increasing air pollution in Ethiopia. Many industries in Ethiopia are categorized on an agricultural basis and account for more than 50% of the country's GDP. Other industries have been found in Addis Ababa and its surrounding areas. Due to its location, it has experienced favorable weather condition that is imaginary for supporting its agricultural activities. Items such as livestock products (eggs, milk, meat, textiles, and leather). It is similarly produced leather goods and processed meat products for the local and export trades. However, its pollution is usually ignored without critical consideration of environmental sustainability and good public health.

The article "Urban Air Pollution and Greenness in Relation to Public Health" was published in 2023. Journal: J Environ Public Health.

The development and expansion of manufacturing industries, construction, and transportation is increasing air pollution without reducing adverse effects [55]. According to World Health Organization (WHO), the 2019 data were classified as “moderate” with an AQI score of 68 and a mean PM_2.5_ count of 20.1 *μ*g/m^3^. This has been a reduction over the earlier years of 2017 and 2018 had been 26.9 *μ*g/m^3^ and 27.1 *μ*g/m^3^, respectively. The 2019 level of pollution made Ethiopia rank 46^th^ as the dirtiest city in the world [43].

### 2.4. Urban Air Quality, Air Quality Index, and Greenness

Currently, greater than 50% of the world's population lives in cities, the majority of which have outdoor air quality standards that fall below those recommended by the World Health Organization for a healthy lifestyle. More than 3 million people die prematurely each year due to air pollution, which is mostly caused by nitrogen dioxide (NO_2_), carbon dioxide (CO_2_), and tiny particles with an aerodynamic diameter of less than 2.5 *μ*m (PM_2.5_). This is more than twice as many people die from traffic accidents [19]. The most effective strategy to enhance the urban air quality is always to reduce pollutant emissions, yet authorities around the world have, almost without exception, struggled to achieve acceptable air quality improvements through emission control strategies alone.

A network of multifunctional greenspace, both urban and rural, is referred to as “green infrastructure” and is capable of providing a variety of environmental and quality-of-life benefits for nearby populations [56]. It may also include “blue infrastructure” such as streams, ponds, canals, and other bodies of water as well as parks, playing fields, other open spaces, woodlands, allotments, and private gardens [57].

Addis Ababa is Ethiopia's largest city and capital and is located in the Horn of Africa. According to a 2017 study, the city has a population of about 5.6 million. At the end of 2020, according to the recommendations of the World Health Organization (WHO), the air quality condition was classified as moderate. The documented value was 76 USAQI with the main pollutant being the fine particulate matter (PM_2.5_) with a concentration of 24 *μ*g/m^3^. WHO specifies a target value of 10 *μ*g/m^3^. 10–12 *μ*g/m^3^ is categorized as “good” and 12.1–35.4 *μ*g/m^3^ is considered “moderate.” The average value of PM_2.5_ in 2019 was 20.1 *μ*g/m^3^ which did not fluctuate much throughout the year.

The article "Urban Air Pollution and Greenness in Relation to Public Health" was published in 2023. Journal: J Environ Public Health.

Greenery gives a semipermeable impact on the flow of pollutants, according to a study by (Tiwary et al., 2011; [58] portrayed that deflecting stream-lines, introduce turbulence and increases dilution, thereby substantially increasing the distance between the source and receptor. Several physical factors, such as plant height and morphology, affect how vegetation interacts with the flow [59]. The spread of air pollutants depends on the vegetation, types of trees, and their height and distance from the source.

### 2.5. Effect of Urban Air Pollution on Health

In an urbanizing world, more and more children are living in cities. Despite various socioeconomic benefits, urban air pollution is related to adverse health effects, mainly due to increased exposure to air pollution [60]. Environmental aspects provide a significant role in increasing the global incidence of respiratory diseases perceived in recent decades [61, 62]. In particular, asthma and nasal conjunctivitis mostly contribute to the global issue of diseases, with a world urban health incidence of schoolchildren of 5–20% and 0.8–39.7%, respectively [63, 64].

Increasing air pollution through rapid urbanization without mitigation has enlarged human exposure to respiratory diseases such as asthma, allergies, fatigue, and bronchitis. [33]. The urban setting and settlement pattern, household density, and green spaces determine the level of air quality and level of exposure [65, 66]. The role of greenery and closeness to green space for school children reduce the exposure level. Respiratory and sensitive symptoms in school children have so far inconsistent results, this is possibly due to changes in exposure timing and green type between different studies [67, 68]. Toxic and unsafe particles (PM_2.5_ and CO_2_) simply enter through the human lung and enter the body's blood vessels [43]. A study by Meo et al. [69] and World Bank [70] portrayed that the effect of the green space environment on air pollutants such as particulate matter PM_2.5_, PM_10_, carbon monoxide (CO), ozone (O_3_), occurrence and death of severe acute respiratory syndrome coronavirus (SARS-CoV-2) in the environmentally highly green urban area is healthier than that of the less-green urban area. The other study reported that the strength of the association observed between PM_2.5_ and mortality decreased as greenness increased [27]. Moreover, the risk of exposure to air pollution in various health results such as hospital admissions [71] and childhood dermatitis was fewer for people living in green areas [72]. Therefore, the benefits of green infrastructure have not only direct benefits but also have indirect effects on health including reduced cardiovascular diseases, asthma, diabetes, and overall mortality as well as reduced heart and lung diseases [14, 60, 73].

The article "Urban Air Pollution and Greenness in Relation to Public Health" was published in 2023. Journal: J Environ Public Health.

Generally, studies focus on the ongoing green to lessen the effects of air pollution on mortality. Compared to those living in a neighborhood with less greenery and residents of poor neighborhoods with high levels of greenery benefited from having more decreased connections between PM_2.5_ and lower mortality [74]. Introducing and implementing pollution-free transportation services, high occupancy vehicles, planned street greenery, and discouraging automobile dependency. This concept helps to improve healthy life and understand better the relationship between air quality, health, and greenness.

## 3. Methods and Materials

This research was conducted in Addis Ababa, the capital city of Ethiopia. The city has become a financial and economic center and is found in the central part of Ethiopia. The city has a medium climate characterized by an urban heat island, glazing buildings, dilapidated settlements, heavy traffic congestion, and many manufacturing industries in and around the city. According to the CSA (2017), the city has about 5.6 million inhabitants. The city has become an economic and diplomatic center of Africa. This has created social and environmental problems such as air pollution, traffic congestion, and depletion of the natural environment for urbanization and industrial development. Therefore, this study was conducted by purposively selecting samples in the city to measure the air quality level of the air tracking device (USAQ Air-visual). The sampling sites have included the manufacturing industry, transportation stations, educational institutions, and residential land use. Quantitative and qualitative research approach had employed to investigate the air pollution level, availability of greenness, and air quality-related health issues. The interview was conducted by industries, the office of the transportation authority, and the environmental protection authority. Transportation stations were taken at the main Arterial Street to measure air quality while manufacturing industry samples were recorded at the city center, intermediate, and expansion area. Measurement of air quality at transportation stations was taken two times during peak and off-peak hours (30 minutes each). The manufacturing industry, residential, and educational institution measured their air quality level one time during working days.

The article "Urban Air Pollution and Greenness in Relation to Public Health" was published in 2023. Journal: J Environ Public Health.

### 3.1. Research Design

The overall research framework was described in (Figure 1).

### 3.2. Sampling and Data Collection

This study was conducted to know air pollution levels and greenness in relation to public health in the city of Addis Ababa. The measurement of air pollution level was taken purposively at eight (8) manufacturing industries and twelve (12) main transportation stations in the city of Addis Ababa by Air visual pro (Figure 2 and Table 1). In this regard, health questionnaire samples were employed for people living in and around the transportation stations and industrial workers. Health questionnaire participants were taken by medical evidence that were affected by respiratory air quality-related diseases which were recorded for a health issue in clinics or hospitals or patient registration number. 480 samples have been purposively taken that have experienced air quality-related health problems in order to analyze the impact of air pollution and greenness in relation to public health. Moreover, an interview was conducted with the concerned body of transportation, environmental protection, and manufacturing industry authority.

### 3.3. Method of Data Analysis

The collected air quality data were converted to excel and analyzed in the mean, percentage, graph, and its relationship between greenness and health. The questionnaire on health was analyzed in a quantitative manner (graphs, percentages, and correlation in a simple linear regression model) and the characteristic of transportation stations, industries, and spatial coverage of greenness and land use were analyzed in the qualitative method. Therefore, those data, the interviews, and observations were administered and explored qualitatively; whereas, the data obtained via questionnaires and air tracking devices were interpreted and analyzed quantitatively. Data on air quality were analyzed by busing US air quality index standards (Table 2).

The relationship between a dependent (health) and independent (air quality) involved in simple linear regression is indicated in equations (1) and (2) (Table 3).

(1) $$\begin{array}{c} Y_{1}=a_{1}+b_{1}X_{1}+e\text{.} \end{array}$$

The equation connected the relationship between health and air quality. In this case, *Y*_1_ the dependent variable represents the extent of the relationship between health and air quality, *a*_1_ is the constant intercept that balances the equation, 𝑏_1_ denotes regression coefficients of the independent variables, and *e* denotes the residual error. *X*_1_ (independent variables), i.e., air quality (PM_2.5_, PM_10_, CO_2_, and AQI).

The article "Urban Air Pollution and Greenness in Relation to Public Health" was published in 2023. Journal: J Environ Public Health.

The other relationship was air quality also depends on greenness (availability of trees in the street, commercial, industries, greenery, and parks).

(2) $$\begin{array}{c} Y_{2}=a_{2}+b_{2}X_{2}+e\text{.} \end{array}$$

*Y*_2_ the dependent variable represents air quality, *a*_2_ is the constant intercept that balances the equation, *b*_2_ denotes regression coefficients of the independent variables, *X*_2_ represents the independent variable greenness, and *e* denotes the residual error.

## 4. Result

### 4.1. Characteristics of Sample Respondents

Of the total (480) respondents, 254 (53%) were males while 226 (47%) were females. The composition of age was categorized into five age categories. Below and equal to18 years old child age, 19–29 years old young age (10 years difference), 30–49 years old adult age (20 years difference), 50–64 years old older people (15 years difference), and the last one was greater than or equal to 65 years old (pensioners). The percentages of respondents were arranged in order from the highest number of participants to the lowest age categories. These were ages between 30–49 (38.54%), 19–29 (28.33%), below 18 (24.17%), 50–59 (7.29%) and 65, and above the age (1.46%), respectively.

### 4.2. Air Pollution and Greenness

The air pollution level was recorded by using an air tracking device (air visual pro) at the selected sampling transportation stations and manufacturing. Air quality measurements were performed twice during peak and off-peak hours (Tables 4–6). Greenness was also assessed in the city particularly street trees at the median and on the walkway, trees between buildings in the manufacturing industry, education institutions, and residential sites (Figure 3). Traffic congestion and manufacturing are polluting the city with a high level of emission (Figures 4 and 5). People and concerned bodies have given less awareness to the pollution impacts rather than economic development.

Greenness within the city and surrounding the city boundary is limited except for the preserved Entoto forest. There is no greenness available on many street networks (on sidewalks and medians). Most road networks in the city do not have street trees and greenery. In Addition to this, public space, parks, and green buffers have not been found enough in the city. Public space, parks, and street greenery are left over in relation to design principles, norms, and standards in the city.

The article "Urban Air Pollution and Greenness in Relation to Public Health" was published in 2023. Journal: J Environ Public Health.

This research has found that PM_2.5_ concentrations in Addis Ababa, Ethiopia tended to be higher (range 30.6 *μ*g/m^3^–202.8 *μ*g/m^3^), due to transportation, power in manufacturing, and charcoal for cooking. The result of health exposure to PM_2.5_ has continuously varied in areas with lower air pollution versus those with greater air pollution concentration. Those people who live and work always proximity to transportation stations and the manufacturing industry were more exposed to health risks (i.e., traffic police, street vendors, employee of the manufacturing industry, and labor at freight terminals).

The average air quality concentration in manufacturing industries was higher than 151AQI (red color) (Figure 4) which is unhealthy for everyone.

Street without street greening or mitigation measure has increased air pollution (Figure 6). Vehicles emit pollutants into the surroundings, particularly at peak hour and pedestrians have been exposed to the emission of the vehicle. Distance and source are directly related to exposure. The distance and the source have a direct relationship with exposure. During air quality observation in an air tracking device, when the walkway became wide the exposure to air pollution slightly decreased. If traffic congestion is high, exposure to air pollution also increased. Particulate matter, CO_2,_ and the air quality index showed 45 *μ*g/m^3^, 1800 ppm, and 152AQI, respectively.

### 4.3. Health Effects of Air Pollution

Simple linear regression analysis of air quality-related diseases and air quality at stations.

The correlation between the occurrence of air quality-related health problems, and an air quality index (AQI) on 12 transportation stations showed that *R*^2^ = 95.47% on average concentration, which is a strong positive relationship with one another (Figure 3). In addition, the correlation between the air quality index and air quality-related health problems among manufacturing industry employees was strong (*R*^2^ = 97.28%). This confirmed that the manufacturing industry emits more pollutants than transportation (Figure 7). The occurrence of air quality-related health problems depends on land use type, greeneries, and the time we spent on the source of air pollution.

Health questionnaires were analyzed based on medical evidence from sampling transportation stations and manufacturing industries. CO_2_ does not have direct health effects, the survey on health was estimated by assessing the ambient concentrations of fine particulate matter and AQI, which have been linked to increased cardiopulmonary mortality and various other acute and chronic health problems, such as aggravation of asthma, respiratory symptoms, and an increase in hospital admissions.

The article "Urban Air Pollution and Greenness in Relation to Public Health" was published in 2023. Journal: J Environ Public Health.

Health effects were estimated using a simple linear regression analysis of air pollutants concentration, and the number of hospital visits for respiratory and cardiovascular diseases.

The World Health Organization estimates that PM contributes to the premature death of about 800,000 people in cities each year and 6.4 million lost healthy life spans [16].

Air pollution poses a threat to the health of the global environment, killing an estimated 3 to 7 million people each year. There are many types of air pollution, but particulate matter (PM) air pollution has the greatest impact on the global disease burden [52, 76]. The effects of air pollution on human health are well documented in many epidemiological studies. Exposure increases the risk of lung cancer, heart disease, bronchitis, and other cardio-respiratory diseases.

The outcomes of this study indicated that people with low socio-economic circumstances were more likely to face a double influence of exposure to air pollution at home, work, or commutes. The collected data have specified that air pollution levels at transportation stations regularly exceed the World Health Organization (WHO) guideline level. Further to this, the air pollution level was usually highest during morning and evening peak hours, regularly getting unhealthy levels throughout the day. The level of PM_2.5_ at transportation stations reached between 35.7 to 205 *μ*g/m^3^ and in manufacturing industries 21 to 212 *μ*g/m^3^ (Figure 8). PM_10_ was released from residential cooking sources and power plants, whereas, fine PM_2.5_ came from motor vehicle engines, electricity, and firewood.

### 4.4. Green Infrastructure to Reduce Human Exposure to Air Pollution

Urbanization and growing demand for housing have transformed large areas of numerous cities into an impermeable urban environment with insufficient greenery. Greenness would treat human health, provide social safety, comfortable, and environmental benefits. Strategic distribution of green infrastructure can reduce exposure to air pollution. However, the development of appropriate design guidelines is vital to promote and optimize the benefits of greening, and measuring the socioeconomic and health benefits of green infrastructures is the key to sustainable development. Greening of cities, especially roadside trees and plantation in manufacturing industries to mitigate pollution effects need to be harmonized through scientific evidence and appropriate policies and strategies. However, there is little empirical evidence linking these benefits to the reduction of air pollution from urban vegetation, and great efforts are needed to establish the essential policies, design principles, and implementation guidelines and their spatial distribution [77, 78].

The article "Urban Air Pollution and Greenness in Relation to Public Health" was published in 2023. Journal: J Environ Public Health.

Some residents were not conscious of the concept of urban green infrastructure and its environmental benefits. [79, 80]. They are aware of only recreation and shading. They have no interest to plant and protect and conserve green infrastructure and open space. There are enacted and approved strategies and policies for green infrastructure to implement in the city. None of them have been implemented in the project due to less attention to greenery and poor monitoring and valuation of a green infrastructure project by the concerned body.

They have given more emphasis to road networks, housing, and high-rise condominium building rather than green infrastructure. The available street network, industries, and residential have not sufficient greeneries based on a plan. Major streets and industries are major sources of the emission of pollutants. The prepared structure plan gave more emphasis on greenery and open space in the built-up pattern but did not implement it on the ground. The city administration and investors have given primary concern for high-density development and consume more space for infill development in the city centers by removing open space and greeneries. The demand for housing and commercial buildings is increasing over time. The construction industries are also increasing with higher air pollutant development in the city.

The interactions of green infrastructure and air pollution in the urban landscape are complex and have a positive or negative impact on air quality, depending on the spatial distribution and GI types. The pros and cons clearly show that certain functions of green infrastructure would be sensitive to local ecological and social conditions.

With rapid urbanization, the sustainability of good air quality in urban regions is a great question now and in the future. This study probed the perceptions of travelers, street vendors, drivers, and traffic police regarding air pollution and how they feel about greenness. The distribution and location of green infrastructure based on land use and function were insufficient (Figure 9). Ethiopia has not successfully implemented standards of air pollution limits by concerned social and environmental protection authorities.

There was not sufficient available street greenery or trees on the major street network of Addis Ababa. The street networks are always busy with traffic congestion mainly during morning and evening peak hours. Vehicles spent longer time on the street due to congestion and emit pollution. This interrupts the pedestrian along walkways and passengers on the road. Using alternative transport options and planting street trees based on standard types of trees that are able to absorb pollutants from motor vehicles to minimize the effects of those pollutants from vehicles. Individuals and the city council and professionals are giving more emphasis on housing and manufacturing industries but neglecting greenness and its negative impact. It needs more focus on planning and implementation of green infrastructure and afforestation on the industrial site, gardens in the residential and commercial district, and street greenery on major street networks (Figures 9 and 10). Sufficient implementation and monitoring of greenery will bring healthy living and maintain the environment from urban heat islands, flooding, and acidic rain, good ecological cycle, and reducing exposure to air quality-related diseases.

The article "Urban Air Pollution and Greenness in Relation to Public Health" was published in 2023. Journal: J Environ Public Health.

Greenness and air pollution interacted nonlinearly with mortality. This study suggested that the air pollutants emitted from vehicles on the street would be minimized with greenness and could protect human health (Figure 11). This also increased well-being, greenness, and air pollution and can be used for public health, urban cooling, and preserving the urban environment.

### 4.5. Implementation of Green Infrastructures

Green infrastructure enterprises can be promoted in two ways. The first one is top-down (government led by financial support and regulation), and the second is bottom-up (communities). Both enterprises have their potential and site-specific challenges, connecting to the practical, economic, environmental, and social considerations for a given project. Therefore, proper directives and programs are needed for the effective implementation of a green infrastructure project. It is understood that top-down green infrastructure enterprises can be implemented on a variety of scales and that policies and strategies need to be motivated by local governments.

## 5. Discussion

As a result of this study, it was found that air pollution in the city has been a key health problem. Since a huge number of vehicles and the manufacturing industry are emitting pollutant gases without air pollution mitigation. Deforestation, rapid urbanization, unable to manage green space, unplanned housing construction, and increased impervious surface have been increasing air pollution. Air pollution level is the primary concern in Addis Ababa. Old fleets, traffic congestion, and unmanaged manufacturing industries emit air pollution to the environment and human health. The result has shown that exposure to air quality-related health problems at main public transportation stations was unsafe (Figures 12 and 3). The road condition with low quality without street greeneries contributed to increase air pollution at the stations. The exposure to air quality-related diseases increased when the age increased (Figure 13). It was also observed that traffic congestion is very high at peak hours (7:00 am–9:30 am and 10:00 pm–1:30 pm). Greenness and alternative transportation systems (nonmotorized transport) improve air quality in the urban environment. According to the interview from the concerned body and empirical evidence, most of the vehicles served more than 25 and 30 years. This also played a major role to increase air pollution such as CO_2,_ PM_2.5,_ and CO.

The article "Urban Air Pollution and Greenness in Relation to Public Health" was published in 2023. Journal: J Environ Public Health.

In the survey of this study, the green coverage was insufficient in the city of Addis Ababa particularly street greeneries, public squares, and parks. These are caused due to urban heat islands, air pollution, and air quality-related diseases. 278 (57.92%) among 480 respondents had experienced air quality-related diseases (Table 7). Out of 278 air quality-related diseases people, 137 dropped under the categories of red air quality index which is unhealthy for humans. This requires special concern for the urban environment, air quality-related diseases, urban greeneries that absorb (particulate matter and CO_2_, CO, NO_X_), nonmotorized transportation, and afforestation.

Dry throat, bronchitis, lung cancer, asthma, difficulty in breathing, pneumonia, emphysema, and fatigue were the major air quality-related diseases in the health survey from the sampling transportation stations and manufacturing industries. When the air quality level was high, the exposure to air quality-related diseases was also increased (Table 8).

According to the result, public transit, and walking are the main means of transportation in Addis Ababa, with 30% and 55% modal share, respectively. The roadside walkway is very narrow, uneven, and congested by street vendors with congested pedestrians, and usually, there is no green on the street. This situation exposed people to air pollution from vehicles during traffic congestion. This needs to prioritize greeneries and management tools to minimize vehicles' air pollution and air quality-related diseases in the urban area.

Mitigating air pollution using green infrastructure in streets, green roofs, and trees in the manufacturing industry is essential for health and environmental protection. Though, empirical evidence of greenness's effectiveness in improving air quality is limited.

Researchers and practitioners continue to struggle with determining how and where greenness can improve air quality. The average annual fine particulate matter concentration had been indicated with 52 *μ*g/m^3^, which is more than double the level messaged by WHO.

The article "Urban Air Pollution and Greenness in Relation to Public Health" was published in 2023. Journal: J Environ Public Health.

Green infrastructure, such as trees and green buildings, is important for health, social safety, comfort, and environmental benefits. Urban greening has the potential to create a wide range of health benefits such as reduced respiratory diseases, fatigue, pneumonia, and psychiatric morbidity, and provide multiple environmental benefits. Nevertheless, there were few practical confirmations relating health effects to air pollution protection from urban greenery. Adopting and implementing green buildings, street trees, urban parks, and mixed neighborhood urban green spaces in cities have a major positive impact on reducing exposure to air quality-related diseases, heat, and air pollution. Air pollution concentration versus source distance; trees planted on the sidewalk on the main street need to have sufficient spacing and should be selected trees that sponge pollutants emitted from vehicles. When the pedestrian walkway is wide, it reduces exposure to pollutants since pollution concentration reduces at a longer distance from the source.

Different green types deliver cooling and air pollution mitigation capabilities, and dense multilayers of different plant types improve overall air pollution. Improving air quality and maximizing green spaces; giving priority to green legacy for transportation stations and industrial land use; and integrating green policies with wider health aspects, transports, and land-use integration policy.

The greenness value to human health has positive significance during the recent worldwide pandemic of COVID-19 since the concentrations of pollutants near roads and industry is changing rapidly over space and time.

Studies in developed countries such as Australia, Canada, Spain, Switzerland, and the USA emission level have become higher than in developing countries, but they are managed by greeneries [81–83]. Individuals in developed countries, with good health, continued to live easily with more greenness and comfortably. According to research results available in scientific literature, a 1 m^2^ leaf area can absorb 70 mg of particulate matter per year [84].

The environmentally green space areas offer the community a happy and healthy living environment [85, 86] study showed that the same result provided some evidence of synergies between greenness and air pollution, suggesting that green space planning and air pollution control can jointly improve public health. However, there were some limitations by some of the studies on air pollution and greenness, in a more recent cross-sectional study using various measurements of exposure to greenness found no association between current asthma and residential surrounding greenness when measured through NDVI, and 60% higher prevalence of current asthma was found to be associated with living close to a park (Cilluffo et al., 2018). The result of this study showed respiratory diseases was highly linked with near industry and transportation terminal that has less greenness.

The article "Urban Air Pollution and Greenness in Relation to Public Health" was published in 2023. Journal: J Environ Public Health.

The location, land use function, and type of vegetation are important for the ability to filter air pollution. The most significant impacts of greenness establishment are likely to be during peak hour traffic congestion when the emissions are greatest. Greenness and air pollution have significant effects on mortality and are consistent. It can be difficult to determine effectiveness empirically. However, actions involving GI may be important to health and air quality (for example, planting trees into a street landscape and green roofs and providing public parks which may reduce particulate matter and urban heat islands) and minimize human exposure to air pollution.

## 6. Conclusions and Recommendations

The result of this study indicated that air quality at transportation stations and industries was very unhealthy for vulnerable groups and unhealthy for the general public. Air quality level has shown between 50.13–96.84 *μ*g/m^3^ of PM_2.5_, 645–1764 ppm of CO_2,_ and 137–179 AQI. Beside this, the green coverage in the city such as street greenery, trees between buildings, and parks was insufficient. Of the 480 health questionnaires, 278 (57.92%) were exposed to air quality-related diseases by medical evidence (i.e., asthma, difficulty in breathing, pneumonia, emphysema, and irritation of the eye). Industry workers, street vendors, traffic police, and drivers were the primary exposures. Based on this research, policy should focus on how to promote urban greenness for a more sustainable and healthy life in urban areas. Peoples have to be aware of air pollution and its consequences. This would help in the successful implementation of urban greenness. Since people seem to accept that urban green infrastructure has certain benefits relating to aesthetical and economic benefits rather than purification of urban air pollution. First, remove the primary source of air pollution by replacing alternative energy that has less pollution. Second, manage and minimize air pollution through urban green infrastructure. Therefore, implementing policies and strategies is vital for the successful reduction of urban air pollution related to transportation and manufacturing industries. Urban development policy has to integrate urban growth and air pollution reduction with greenness and ensure sufficient space for sidewalk width, protection of green space, and access to greenery for a sustainable quality of life. Transportations and industries' air pollution have given the least attention in the capital city of Ethiopia, Addis Ababa in particular, and developing cities worldwide in general. This study indicated the initial concept about the impact of urban air pollution on health and greenness for minimizing air pollutants and improving human health. There was a limitation on the measurement of air quality. It has taken only peak hours (7:30–9:00 am and 5:00–7:30 pm) and off-peak hours (9:30 am–4:30 pm). This needs further investigation of urban air pollution related to time and space 24 hours a day at industries, transportation stations, and residential sites.

The article "Urban Air Pollution and Greenness in Relation to Public Health" was published in 2023. Journal: J Environ Public Health.

## Figures and Tables

**Figure 1:** Research design.

**Figure 2:** Location of the study and sample dissemination of transportation stations and industries.

**Figure 3:** number of incidences of air quality-related health problems and AQI at stations.

**Figure 4:** Average air quality index in manufacturing industries.

**Figure 5:** Air quality by the speed of a car on the road (A to F level of service).

**Figure 6:** Vehicles air pollution without street greeneries.

**Figure 7:** Number of incidences of air quality-related health problems and AQI at manufacturing.

**Figure 8:** Particulate matter at peak hour and off-peak hour.

**Figure 9:** Built-up and greeneries coverage in the city of Addis Ababa.

**Figure 10:** Intervention area and proposed land use with road network and greenery.

**Figure 11:** Street greenery on major roads to reduce air pollutants from vehicles.

**Figure 12:** Average air quality index at transportation stations.

**Figure 13:** Frequency of clinic visits for air quality-related health issues in the past time.

**Table 1:** Sample size, location, and target populations for health questionnaire.

No	Name	Sample site	Sample size	Targeted population
1	Transportation stations	Sidist Kilo	24	(i) Drivers, (ii) traffic policies, (iii) passengers, (iv) transport coordinators, (v) street vendors, (vi) shoeshines, (vii) street sweepers, and (viii) residents nearby the station within 500 meters
		Menelik II Square	24	
		Autobus Tera	24	
		Torhayloch	24	
		Mexico	24	
		Megenagna	24	
		Ayat	24	
		Ayer Tena	24	
		Bole Deldy	24	
		Haile Garment	24	
		Adey Abeba	24	
		Kality	24	

2	Manufacturing industries	Jemo Glass Industry	24	(i) Industry workers and (ii) residents around the industry
		Bole Lemi Industry	24	
		Kality Industry Park	24	
		Sar-bet Medium Industry	24	
		Gotera Moha Industry	24	
		Pacific Industry	24	
		Mesalemia Industry	24	
		Star Soap Detergent Industry	24	

Total		20	480	Air quality-related diseases

The article "Urban Air Pollution and Greenness in Relation to Public Health" was published in 2023. Journal: J Environ Public Health.

**Table 2:** Air quality categories, standards, and health messages.

AQI value	AQI color	PM_2.5_ (*μ*g/m^3^)	PM_10_ (*μ*g/m^3^)	CO_2_ (ppm)	AQI category and health messages
0–50	Green	0–12.4	0–54	<700	Good
51–100	Yellow	12.5–35.4	55–154	701–1,000	Moderate
101–150	Orange	35.5–65.4	155–254	1,001–1,500	Unhealthy for sensitive groups
151–200	Red	65.5–150.4	255–354	1,501–2,500	Unhealthy
201–300	Purple	150.5–250.4	355–424	2,501–5,000	Very unhealthy
301+	Maroon	250.5+	425+	5001+	Hazardous

Source: [75].

**Table 3:** Dependent and independent variables involved in the simple linear regression model.

Variables	Definition	Unit	Variable types
Dependent (*y*)	Health	—	Nominal
	Air quality	—	Continuous

Independent (*x*)	Carbon di oxide (CO_2_)	Ppm	Continuous
	Air quality index (AQI)	—	Continuous
	Particulate matter (PM_2.5_, PM_10_)	*μ*g/m^3^	Continuous
	Speed of vehicles on the road	km/h	Continuous
	Availability of trees and green space on the road network and park	(No, yes)	Binary
	Population density	pop/hectare	Continuous
	Land use type	—	Nominal

	Foot traffic	p/min/feet	Continuous

**Table 4:** Average air quality index in manufacturing industries.

Manufacturing	PM_2.5_ (*μ*g/m^3^)	PM_10_ (*μ*g/m^3^)	CO_2_ (ppm)	AQI	Temperature (C°)	Humidity (%)
Jemo Glass Industry	83.71	159.22	1028.01	174	24.5	45.3
Bole Lemi Industry	80.63	127.31	1307.54	158	22.8	48.7
Kality Industry Park	86.42	164.34	1538.16	176	25.6	43.9
Sar-bet Industry	89.38	173.28	1961.84	175	21.7	46.2
Gotera Moha Industry	79.25	151.22	1451.91	151	21.6	51.3
Pacific Industry	81.34	148.91	1287.35	157	23.5	47.6
Mesalemia Storage	96.84	187.62	1764.73	179	22.5	50.7
Star Soap Detergent Industry	78.89	154.64	1524.53	152	26.7	45.4

**Table 5:** Peak hour average air quality level at transportation stations.

Transportation stations	PM_2.5_ (*μ*g/m^3^)	PM_10_ (*μ*g/m^3^)	CO_2_ (ppm)	AQI	Temperature (C°)	Humidity (%)
Kality	68.12	109.81	1167.25	156	21.6	50.5
Adey Abeba	85.09	128.65	1407.41	162	24.2	54.6
Haile Garment	71.94	122.54	1226.54	150	23.1	53.4
Bole Deldy	87.17	129.65	1836.49	171	19.9	52.9
Sidist Kilo	71.52	120.87	798.24	152	18.3	58.7
Ayat	78.01	125.34	834.47	159	20.8	54.8
Megenagna	91.38	148.65	1875.62	170	22.5	55.7
Mexico	87.69	130.47	1563.12	160	23.6	57.3
Torhayloch	89.01	137.54	1547.28	168	24.9	54.4
Ayer Tena	79.14	127.31	1421.95	150	24.7	53.7
Autobus Tera	93.61	152.61	1765.73	172	23.1	54.1
Menelik II Square	90.89	140.31	1498.46	169	20.6	55.4

**Table 6:** Off-peak hour average air quality level at transportation stations.

Transportation stations	PM_2.5_ (*μ*g/m^3^)	PM_10_ (*μ*g/m^3^)	CO_2_ (ppm)	AQI	Temperature (C°)	Humidity (%)
Kality	50.46	76.31	561	138	25.3	37.6
Adey Abeba	72.34	115.35	679	153	26.6	35.6
Haile Garment	67.64	109.24	552	146	25.9	38.3
Bole Deldy	79.12	130.53	588	165	22.4	34.9
Sidist Kilo	56.43	87.31	542	143	25.6	34.1
Ayat	70.24	103.22	602	148	24.7	32.6
Megenagna	75.64	120.64	698	165	25.1	35.7
Mexico	62.64	105.42	679	154	23.5	37.1
Torhayloch	61.51	103.62	597	152	25.7	29.4
Ayer Tena	50.13	75.31	645	137	26.8	30.7
Autobus Tera	77.16	128.54	781	166	24.3	33.7
Menelik II Square	70.56	106.45	551	160	21.5	34.3

The article "Urban Air Pollution and Greenness in Relation to Public Health" was published in 2023. Journal: J Environ Public Health.

**Table 7:** Air quality index versus clinic visited for air quality-related diseases.

Air quality index	Visited clinics/hospitals		Total	Percent of air quality-related diseases (%)	Percent of nonair quality-related diseases (%)
	Air quality-related diseases	Nonair quality-related diseases			
0–50 (green)	8	81	22	2.88	40.10
51–100 (yellow)	41	57	91	14.75	28.22
101–150 (orange)	92	50	149	33.09	24.75
151–200 (red)	137	14	218	49.28	6.93
201–300 (purple)	0	0	0	0.00	0.00
301–500 (maroon)	0	0	0	0.00	0.00

Total	278	202	480	57.92	42.08

**Table 8:** Characteristics of transportation stations and traffic conditions.

Sample site	Cars traffic (km/h)	Availability of trees	Density (pop/ha)	Land use	Foot traffic (p/min/feet)	Time
Kality	43.1–54.4	No	350	Commercial	11–15	5:00 pm
Adey Abeba	0–25	No	436	Mixed	>16	8:00 am
Haile Garment	33.6–43	No	376	Industry	11–15	6:00 pm
Bole Deldy	33.6–43	Yes	394	Commercial	>16	6:00 pm
Sidist Kilo	43.1–54.4	Yes	384	Service	>16	5:00 pm
Ayat	54.5–67	No	502	Residential	11–15	8:00 am
Megenagna	0–25	No	391	Commercial	>16	5:00 pm
Mexico	0–25	No	406	Commercial	>16	8:00 am
Torhayloch	25.1–33.5	No	324	Special function	11–15	7:00 am
Ayer Tena	43.1–54.4	No	409	Mixed	>16	8:00 am
Autobus Tera	0–25	No	338	Commercial	>16	6:00 pm
Menelik II Square	25.1–33.5	Yes	387	Administration	11–15	5:00 pm

## Data Availability

The data that supports the findings of this study can be obtained from the corresponding author.
